The article "Higher Rumination Tendency Is Associated with Reduced Positive Effects of Daily Activity Participation in People with Depressive Disorder" was published in 2022. Journal: Occup Ther Int.

# Higher Rumination Tendency Is Associated with Reduced Positive Effects of Daily Activity Participation in People with Depressive Disorder

**DOI:** 10.1155/2022/1409320

**Published:** 2022-03-17

**Authors:** Lin-Jye Huang, Chinyu Wu, Hsin-Hsiu Essential Yeh, Pei-Shan Huang, Yi-Hong Yang, Yung-Chun Fang, Chien-Te Wu

**Affiliations:** ^1^Department of Psychiatry, Taipei City Hospital Yangming Branch, Taipei, Taiwan; ^2^School of Occupational Therapy, College of Medicine, National Taiwan University, Taipei, Taiwan; ^3^Department of Occupational Therapy, School of Health Science, Winston-Salem State University, Winston-Salem, North Carolina, USA; ^4^Faculty of Rehabilitation Medicine, University of Alberta, Edmonton, Alberta, Canada; ^5^Planning Division, Bureau of National Health Insurance, Taipei, Taiwan; ^6^International Research Center for Neurointelligence (WPI-IRCN), The University of Tokyo Institutes for Advanced Study (UTIAS), The University of Tokyo, Tokyo, Japan

## Abstract

**Objectives:**

Rumination, a response style characterized by self-reflection loops of negative thoughts, tends to exacerbate depressive symptoms and may impair daily functional behaviors of individuals with depression. However, the specific impacts of rumination on activity participation remain unclear. The current study was aimed at examining the differences in daily activity participation profiles between clinically depressed people with higher versus lower rumination tendencies, with the hope to provide insightful suggestions for improving the quality of life of ruminative individuals with major depression.

**Methods:**

We recruited 143 participants with a depression-related diagnosis from psychiatric daycare centers or clinics and analyzed the differences in activity participation profiles between individuals with higher versus lower rumination tendencies.

**Results:**

Although compared to those with lower rumination tendencies, participants with higher rumination tendencies spent a longer time in activity participation; they experienced lower participation quality during these activities. Furthermore, their activity participation was primarily motivated by meeting others' expectations rather than self-interest. They also misattributed participation restriction to “lack of family support,” indicating that the unhealthy rumination pattern might be the cause of their lack of positive feelings from engaging in meaningful daily activities.

**Conclusions:**

The current results suggest that the unhealthy motivation behind activity participation seems to be an important factor that decreases the quality of participation in individuals with higher rumination tendency. Establishing a healthy motivation for activity participation is therefore critical for improving their quality of participation. As an initial step, OT interventions could put a focus on helping them clarify and escape from the source of negative rumination cycles that impede their positive feeling of activity participation.

The article "Higher Rumination Tendency Is Associated with Reduced Positive Effects of Daily Activity Participation in People with Depressive Disorder" was published in 2022. Journal: Occup Ther Int.

## 1. Introduction

Depressive disorders are a common mental illness affecting almost 300 million people worldwide, causing a tremendous global burden [1]. Depression typically poses threats to people by affecting their mood, behavior, cognition, and somatic conditions, which leads to functional impairments in physical activity and social roles, and less participation in daily life [2–4]. The illness duration and severity of depression vary across the population, with some show remission after several days, whereas others remain severe from months to years [5, 6]. Trait rumination has been proposed to be one factor that accounts for the heterogeneity of depression [7].

According to the response styles theory of depression [7], rumination refers to repetitive and passive thinking loops about the individual's depressive symptoms and the possible causes and consequences. This type of depressive rumination prevents an individual from participating in pleasant activities to escape from dysphoric moods or take actions in response to stressful life events. It can thus prolong the duration and increase the severity of depression. Trait rumination may also result in many harmful outcomes, including depressive symptoms, negatively biased thinking, poor problem-solving, impaired motivation and inhibition of instrumental behavior, impaired cognition, and increased stress levels [8]. Moreover, rumination is detrimental to an individual's occupational performance, such as attention span in academic tasks, problem-solving abilities, interpersonal relationships, and social functioning [9–11]. For evaluating rumination levels, the ruminative response scale (RRS) [12] is a well-known instrument that has been validated across different cultures and populations [13–15]. However, the RRS has been questioned to contain several nonrumination-specific items [16, 17]. Thus, Treynor et al. [18] removed 12 confounding items and revalidated the brief RRS, yielding a two-factor structure, “reflection” and “brooding.” “Reflection” refers to a neutral manner consideration about the ways to cope with problems, whereas “brooding” refers to pondering moodily or anxiously about the negative issues related to oneself, including self-criticism. Notably, *brooding*, representing pure ruminative responses (e.g., “What am I doing to deserve this?”), shows a higher correlation with depression than *reflection*.

The article "Higher Rumination Tendency Is Associated with Reduced Positive Effects of Daily Activity Participation in People with Depressive Disorder" was published in 2022. Journal: Occup Ther Int.

The World Health Organization [19] proposed a common framework, the *International Classification of Functioning, Disability, and Health* (ICF), to describe health-related status in humans that shifts the attention from a pathological viewpoint to an integrative and interactive perspective, emphasizing the importance of “activity” and “participation.” In line with the new focus of ICF, previous studies have shown that activity participation may be an effective solution to reduce rumination and help recover from depressed mood or improve the subjective quality of life [20–23]. Also, Huang et al. [13] demonstrated that individuals with higher depressive rumination tendencies showed poorer subjective feelings (e.g., sense of involvement and self-worth) of daily activity participation than those with lower depressive rumination tendencies. However, little is known about how levels of trait rumination affect an individual's participation profile in everyday activities. Such knowledge will provide suggestive evidence to guide our intervention strategy to help people with higher rumination tendency to improve their quality of activity participation. Therefore, in this study, we examined and compared the differences in the participation profiles and participation restrictions of daily activities between individuals with higher versus lower rumination in the clinically depressed population, intending to provide translational information for practical intervention in mental health.

## 2. Materials and Methods

### 2.1. Participants

The current study used a cross-sectional design and questionnaire-based evaluations to investigate the relationship between participants' rumination tendency and their health-related outcomes. We recruited study participants from clinics or day treatment programs of multiple hospitals in Taiwan. The screening criteria included (A) age between 18 and 65 years and (B) one of the following the *Diagnostic and Statistical Manual of Mental Disorders*, fourth edition, Text Revision (DSM-IV-TR) [2] diagnosis: major depression, bipolar I with a recent episode of depression, bipolar II, and dysthymic disorder. The study protocol was approved by the Institutional Review Board of the Taipei City Hospital (No. TCHIRB-960109-E). Before participation, each participant was debriefed, by a trained assistant, about the study purpose, measurements, required time to filling in the questionnaires (about 30 minutes), the confidentiality agreement, and the right to terminate at any time. After signing the informed consent, each participant was tested in a quiet, isolated room or space at the participating departments, either individually or in a small group. All participants were provided with standardized instructions when conducting the tests.

The article "Higher Rumination Tendency Is Associated with Reduced Positive Effects of Daily Activity Participation in People with Depressive Disorder" was published in 2022. Journal: Occup Ther Int.

### 2.2. Research Instruments

#### 2.2.1. Ruminative Response Scale-Chinese version (RRS-C)

The RRS-C contained 22 items to measure ruminative response style. The respondents self-reported and used a four-point scale to rate their responses to the depressed moods. Huang et al. [13] translated and validated the Chinese version of RRS, and the results have shown good validity and reliability. The RRS-C yielded three factors, including “symptom-based” (e.g., “Why do I always react this way?”), “isolation/introspection” (e.g., “Go away by yourself and think about why you feel this way”), and “self-focus” (e.g., “Think about a recent situation, wishing it would have gone better”). The brief RRS-C yielded two factors, “brooding” and “reflection.” Cronbach's alpha values for the factors in RRS-C or brief RRS-C ranged from acceptable (0.71) to excellent (0.92). Furthermore, Huang et al. adopted standard reference BDI-II score 31 to find that the “brooding” subscore 12 in the brief RRS-C was the optimal cutoff point to determine the higher vs. lower rumination tendency (for details, please see their original works in reference [13]).

#### 2.2.2. Beck Depression Inventory-II (BDI-II) Chinese version

BDI-II is a four-point Likert scale (from 0 to 3 by the severity of symptoms) with 21 self-reported inventory items, a reliable instrument to measure the severity of depression from teenagers to adults [24]. BDI-II has been revised since 1994 for recruiting several elements which contained the principles of the *Diagnostic and Statistical Manual of Mental Disorders*, fourth edition (DSM-IV) [25], including dysphoria, worthlessness, insomnia, poor concentration, appetite, and energy [26]. The Chinese version of the BDI-II had good reliability and validity on psychiatric outpatients. The BDI-II score 31 is the bias-corrected threshold score for identifying people with or without severe depression in Taiwan [27].

#### 2.2.3. Activity Participation and Restriction Questionnaire (APRQ)

APRQ was developed to measure activity participation and participation restriction for community-dwelling people with severe mental illness [28]. The respondents are encouraged to provide up to five meaningful activities they regularly attend within the past two months, followed by filling out each activity's participation profile. The profile includes participation duration, frequency, coparticipants, place, purpose, and subjective feelings: “sense of involvement,” “positive affects,” “negative affects,” and “self-worth.” Meanwhile, the respondents are also encouraged to list up to five activities they perceive as being restricted from participation, elaborating reasons for such restriction and rating their subjective feelings regarding “expected involvement” and “negative effects due to restriction.” The reliability and validity of APRQ are acceptable on the sample of 346 community-dwelling individuals with severe mental illness in Taiwan [29].

The article "Higher Rumination Tendency Is Associated with Reduced Positive Effects of Daily Activity Participation in People with Depressive Disorder" was published in 2022. Journal: Occup Ther Int.

### 2.3. Statistical Analyses

We used the Statistical Package of the Social Science software version 21.0 for Windows (SPSS, Chicago, Illinois, USA) to analyze data. We applied the optimal cutoff score of 12 on the “brooding” factor of the brief RRS-C to divide the participants into two groups with higher rumination tendency (HR) and lower rumination tendency (LR), respectively, in this study. Then, we referred to the principles of activity classification on ICF [19] and the study of Linden et al. [30] to recode the activities provided by the subjects in the APRQ into different activity categories. Finally, we used the Wilcoxon rank-sum test for examining continuous variables and the Fisher's exact test for categorical variables of the participants' demographical characteristics, activity participation, and participation restriction profiles between HR and LR groups.

## 3. Results

This study enrolled 143 Taiwanese participants (102 females and 41 males) with a mean age of 44 years old (standard deviation = 9.0 and range = 19–60 years).  Table 1 summarizes the demographical data of both higher and lower rumination tendency groups (denoted as HR and LR, respectively). First, HR had a significantly higher percentage of “females” with younger age and more severe depressive symptoms than LR. Meanwhile, in terms of the classification of diagnosis, HR had a marginally higher percentage of “bipolar II” than LR (*p* = 0.051); instead, LR had a significantly higher percentage of “major depression” than HR. Furthermore, in marriage status, HR had a higher rate of “divorced” than LR, but LR had a higher rate of “married” than HR. Moreover, in religious beliefs, HR had a higher rate of “none” than LR, but LR had a higher rate of “Buddhism” than HR. Finally, in the supporting system, HR had a higher percentage of “from religion” than LR but a lower percentage of “from family” rate than LR. Thus, the two groups differed remarkably in the gender ratio, age, depression severity, diagnosis classifications, marriage status, religious beliefs, and supporting systems.

Table 2 summarizes the differences in the profiles of activity participation between HR and LR. HR showed substantially higher activity participating hours but a lower sense of involvement than LR. Additionally, HR had a higher percentage of “meeting other's expectations” than LR for activity participation purposes. Instead, LR had a higher percentage of “like being with people” than HR. Thereby, the two groups differ significantly in participating hours, purposes, and sense of involvement, but not in the activity types, frequency, numbers of coparticipants, and participation settings.

The article "Higher Rumination Tendency Is Associated with Reduced Positive Effects of Daily Activity Participation in People with Depressive Disorder" was published in 2022. Journal: Occup Ther Int.

Table 3 reveals the differences in the profiles of participation restriction between HR and LR. The two groups showed insignificantly different activity types of restriction participation, except HR, which demonstrated a slightly higher “vocational activity” rate than LR (*p* = 0.045). Generally, the two groups differed insignificantly on the subjective feelings of expected involvement and adverse affections due to restriction. Notably, the two groups showed significant differences in the distribution of the perceived reasons for participation restriction. HR had a higher rate of “without family's support” than LR, while LR had a higher rate of “poor health status” than HR.

## 4. Discussion

The current study examined the participation profiles of the most critical and meaningful daily activities between clinically depressed individuals with high and low rumination tendencies. Our study results showed that the clinically depressed individuals with higher rumination tendencies are characteristically different from those with lower rumination tendencies regarding gender, age, marital status, religious beliefs, and supporting systems. The features for people with higher rumination tendencies may include female [31], younger age [32], diagnosis of bipolar disorder [33], unsatisfied marriage status [34], fewer needs for religious beliefs [35], and less perceived social support [36, 37]. This consistency suggests that our study results on activity participation profiles may reflect more transparent and authentic outlines in their life context.

Compared to those with higher rumination tendency, individuals with lower rumination tendency showed lower severity of depressive symptoms and their meaningful daily activity participation was mainly motivated by “like being with others,” indicating a friendly interpersonal relationship or network may help facilitate their intrinsic motivation for activity participation. In contrast, individuals with higher rumination tendency showed severer depressive symptoms. Their activity participation was mostly motivated by “meeting other's expectations.” It seems that they demonstrated non-self-motivated behaviors to participate in meaningful daily activities, as manifested by longer activity time but with a lower sense of engagement and stressful interpersonal relationships. This result also indicates that the vicious cycles of daily participation still exist and worsen the prognosis of depression. In the core philosophy of occupational therapy, occupation may include significant habits, routines, rituals, and roles that form an individual's daily life [38]. Participating in meaningful occupations, primarily work and leisure, is crucial to positively enhance self-identity, health, well-being, and everyday life goals [3, 39–41]. However, our results contradicted this proposal, revealing that clinically depressed individuals with higher rumination did not seem to gain benefit from participating in their essential and meaningful daily activities. Future studies are needed to validate our suggestion that they may need professional interventions to improve their activity participation quality through modifying their daily activity participation profiles as a starting point.

The article "Higher Rumination Tendency Is Associated with Reduced Positive Effects of Daily Activity Participation in People with Depressive Disorder" was published in 2022. Journal: Occup Ther Int.

Moreover, in terms of the participation restriction, although the individuals with higher rumination tendency demonstrated a remarkably higher restraint from “vocational activity” than those with lower rumination tendency, they did not feel much disappointment from such restriction. In addition, they consider such participation restriction mainly resulted from “lack of family's support.” According to McIntosh et al. [42], the depressed people with higher rumination tendencies tend to link unexpected negative outcomes in everyday life adversely (e.g., lack of family support or worse interpersonal relationships) to the long-term negative consequences of life span (e.g., no hope in looking for an excellent job or deserving a better life). That means when the hopeless feeling is triggered by the combined effects between rumination and inappropriate interpretations of the adverse or stressful life events, it may lead to severer rumination and depressive symptoms [43]. Therefore, disentangling such arbitrary and incorrect causal links is critical to help provide a way out of ruminative thinking [44]. Based on this viewpoint, psychoanalytical approaches such as expressive activities with inner thought reflection and analysis have been strongly advocated to help alleviate rumination and depressive symptoms [21, 45, 46]. That explains why we rarely found the participants with higher rumination tendencies conducted similar emotionally expressive activities in this study.

From the emotion regulation perspective, rumination is not a healthy strategy for relieving depressive moods as it is incredibly exhausting and usually leads to adverse consequences [47]. In contrast, some other positive emotion regulation strategies, such as reappraisal, problem-solving, and acceptance, may reduce the severity of depression [48]. Accordingly, it is necessary to incorporate these better approaches into the intervention programs to help individuals with higher rumination reestablish their meaning of life and rearrange daily activities priorities. For example, expressive writings could help them clarify incorrect associations between causes and effects to prevent unhealthy rumination cycles.

The article "Higher Rumination Tendency Is Associated with Reduced Positive Effects of Daily Activity Participation in People with Depressive Disorder" was published in 2022. Journal: Occup Ther Int.

Please note that there were four limitations in the current study. First, our sample size is relatively small, and thus, the findings should be cross-validated in a larger sample size. Second, our study sample may not be well-representative of people with major depressive disorder because we also recruited bipolar disorder or dysthymic disorder. Thus, this study's findings should be applied with caution to individuals with different types of depression. Third, we excluded the profiles of the second and third activities in activity participation and participation restriction, respectively, in APRQ to prevent bias due to too much missing data. Fourth, the current study was all based on self-administered assessments which may limit the scopes and discussions of the related issues. Future researches may consider developing and applying more objective measurements to conduct validation between variables.

This study brings in the theoretical perspective of rumination, which may deepen practitioners' knowledge of depression. This study indicated that individuals with higher rumination tendencies demonstrate worse activity participation profiles than those with lower rumination tendencies. This finding may lead to more effective intervention guidelines for reducing rumination and enhancing daily activity participation in people with depression.

## 5. Conclusion

In summary, our results confirm that the features for clinically depressed individuals with higher rumination tendency might include females, younger age, diagnosis of bipolar disorder, unsatisfied marriage status, fewer needs for religious beliefs, and less perceived social support. Moreover, our findings clearly outline that they tend to spend a long time doing their most important daily activities, motivated mainly by meeting others' expectations but experienced less involvement and fewer family supports while participating in these activities. Therefore, it is critical to help them reestablish individualized life goals as healthier motivations for activity participation, leading to a more satisfactory experience of their everyday lives.

## Figures and Tables

**Table 1:** A summary of the demographic and clinical characteristics of participants in the current study (*N* = 143).

Variable	Higher rumination	Lower rumination	Total	*p*
Number of subjects (*n*)	88 (61.54%)	55 (38.46%)	143 (100%)	
Gender				<0.001^∗∗∗^
Female	72 (81.82%)	30 (54.55%)	102 (71.33%)	
Male	16 (18.18%)	25 (45.45%)	41 (28.67%)	
Age (years)	42.58 ± 8.97	45.73 ± 9.31	43.79 ± 9.20	0.046^∗^
Onset age of illness (years)	36.35 ± 8.12	38.47 ± 9.89	37.13 ± 8.83	0.182
Duration of illness (years)	6.47 ± 4.70	7.16 ± 5.02	6.73 ± 4.82	0.414
BDI-II	41.54 ± 7.35	28.15 ± 15.25		<0.001^∗∗∗^
Diagnosis				0.043^∗^
Major depression	37 (42.05%)	33 (60.00%)	70 (48.95%)	0.041^∗^
Bipolar I with most recent episode of depression	16 (18.18%)	5 (9.09%)	21 (14.69%)	0.153
Bipolar II	22 (25.00%)	6 (10.91%)	28 (19.58%)	0.051
Dysthymic disorder	13 (14.77%)	11 (20.00%)	24 (16.78%)	0.492
Education				0.232
Elementary school	3 (3.45%)	7 (12.73%)	10 (7.04%)	0.046^∗^
Junior high school	8 (9.20%)	5 (9.09%)	13 (9.15%)	1.000
Senior high school	38 (43.68%)	22 (40.00%)	60 (42.25%)	0.729
College	38 (43.68%)	21 (38.18%)	59 (41.55%)	0.601
Missing	1	0	1	
Marriage				0.004^∗∗^
Unmarried	21 (24.14%)	11 (20.00%)	32 (22.54%)	0.681
Married	37 (42.53%)	37 (67.27%)	74 (52.11%)	0.006^∗∗^
Separated	5 (5.75%)	0 (0.00%)	5 (3.52%)	0.156
Divorced	20 (22.99%)	3 (5.45%)	23 (16.20%)	0.005^∗∗^
Widower/widow	4 (4.60%)	4 (7.27%)	8 (5.63%)	0.711
Missing	1	0	1	
Religion				0.006^∗∗^
None	35 (39.77%)	13 (23.64%)	48 (33.57%)	0.046^∗^
Christianity	13 (14.77%)	2 (3.64%)	15 (10.49%)	0.080
Buddhism	19 (21.59%)	24 (43.64%)	43 (30.07%)	0.008^∗∗^
Taoism	21 (23.86%)	16 (29.09%)	37 (25.87%)	0.434
Economic source				0.558
Earned by self or saving	41 (53.25%)	22 (44.90%)	63 (50.00%)	0.465
Supported by family	34 (44.16%)	25 (51.02%)	59 (46.83%)	0.470
Supported by low-income subsidies from government	0 (0.00%)	1 (2.04%)	1 (0.79%)	0.389
Supported by disability benefits from government	1 (1.30%)	1 (2.04%)	2 (1.59%)	0.389
Others	1 (1.30%)	0 (0.00%)	1 (0.79%)	1.000
Missing	11	6	17	
Supporting system				0.002^∗∗^
From religion	15 (17.05%)	2 (3.92%)	17 (12.23%)	0.030^∗^
From family	29 (32.95%)	33 (64.71%)	62 (44.60%)	<0.001^∗∗∗^
From medical staffs	25 (28.41%)	7 (13.73%)	32 (23.02%)	0.060
From friends	19 (21.59%)	9 (17.65%)	28 (20.14%)	0.825
Missing	0	4	4	

The sample statistics presented in this table were mean ± standard deviation (SD) for continuous variables and frequency (percentage, %) for categorical variables. The listed *p* values of statistical tests were calculated using the Wilcoxon rank-sum test for continuous variables and the Fisher's exact test for categorical variables.

^∗^ *p* < 0.05, ^∗∗^*p* < 0.01, and ^∗∗∗^*p* < 0.001.

The article "Higher Rumination Tendency Is Associated with Reduced Positive Effects of Daily Activity Participation in People with Depressive Disorder" was published in 2022. Journal: Occup Ther Int.

**Table 2:** The differences in participation profiles of the most meaningful activities between participants with higher vs. lower rumination tendency.

Variable	Higher rumination	Lower rumination	Total	*p*
Types of participation				0.398
Cultural activity	17 (19.32%)	9 (16.98%)	26 (18.44%)	0.825
Social activity	5 (5.68%)	1 (1.89%)	6 (4.26%)	0.410
Hobby activity	8 (9.09%)	5 (9.43%)	13 (9.22%)	1.000
Physical activity	11 (12.50%)	12 (22.64%)	23 (16.31%)	0.157
Health maintenance	10 (11.36%)	9 (16.98%)	19 (13.48%)	0.446
Home activity	11 (12.50%)	8 (15.09%)	19 (13.48%)	0.800
Vocational activity	26 (29.55%)	9 (16.98%)	35 (24.82%)	0.110
Missing	0	2	2	
Frequency of participation				0.155
Less than once a month	2 (2.27%)	0 (0.00%)	2 (1.43%)	0.530
Once a month	1 (1.14%)	0 (0.00%)	1 (0.71%)	1.000
Twice to thrice a month	3 (3.41%)	0 (0.00%)	3 (2.14%)	0.295
Once a week	16 (18.18%)	6 (11.54%)	22 (15.71%)	0.345
Twice to thrice a week	8 (9.09%)	9 (17.31%)	17 (12.14%)	0.184
Quartic to sextic a week	8 (9.09%)	9 (17.31%)	17 (12.14%)	0.184
Once a day	39 (44.32%)	17 (32.69%)	56 (40.00%)	0.213
More than twice a day	11 (12.50%)	11 (21.15%)	22 (15.71%)	0.230
Missing	0	3	3	
Co-participants of participation				0.917
Alone	50 (57.47%)	27 (54.00%)	77 (56.20%)	0.724
Family	13 (14.94%)	7 (14.00%)	20 (14.60%)	1.000
Ward mates	4 (4.60%)	3 (6.00%)	7 (5.11%)	0.706
Medical staffers	0 (0.00%)	0 (0.00%)	0 (0.00%)	—
Colleagues	9 (10.34%)	6 (12.00%)	15 (10.95%)	0.770
Friends/classmates	10 (11.49%)	5 (10.00%)	15 (10.95%)	0.572
Others	1 (1.15%)	2 (4.00%)	3 (2.19%)	0.138
Missing	1	5	6	
Settings of participation				0.976
Home	31 (35.23%)	21 (40.38%)	52 (37.14%)	0.589
Hospital	9 (10.23%)	6 (11.54%)	15 (10.71%)	0.785
Market/department store	2 (2.27%)	1 (1.92%)	3 (2.14%)	1.000
Company/workplace	16 (18.18%)	9 (17.31%)	25 (17.86%)	1.000
Park/play ground	8 (9.09%)	6 (11.54%)	14 (10.00%)	0.211
Church/Temple	5 (5.68%)	2 (3.85%)	7 (5.00%)	0.196
School/classroom	10 (11.36%)	3 (5.77%)	13 (9.29%)	0.099
Others (e.g., swimming pool)	7 (7.95%)	4 (7.69%)	11 (7.86%)	0.956
Missing	0	3	3	
Purposes of participation				<0.001^∗∗∗^
For economic reasons	18 (21.43%)	5 (10.00%)	23 (17.16%)	0.246
Like being with people	1 (1.19%)	7 (14.00%)	8 (5.97%)	0.013^∗^
Meeting other's expectations	20 (23.81%)	0 (0.00%)	20 (14.93%)	<0.001^∗∗∗^
Own responsibility	15 (17.86%)	13 (26.00%)	28 (20.90%)	0.135
Relaxing body and mind	22 (26.19%)	18 (36.00%)	40 (29.85%)	0.249
Others (e.g., religious belief)	8 (9.52%)	7 (14.00%)	15 (11.19%)	0.086
Missing	4	5	9	
Participation hours	4.99 ± 4.01	3.13 ± 2.47	4.29 ± 3.62	<0.001^∗∗∗^
Coparticipants' numbers	2.78 ± 6.84	2.76 ± 5.10	2.77 ± 6.25	0.989
Sense of involvement	2.36 ± 0.55	2.55 ± 0.52	2.43 ± 0.55	0.041∗
Positive affection	2.27 ± 0.52	2.37 ± 0.57	2.31 ± 0.54	0.272
Negative affection	1.51 ± 0.57	1.49 ± 0.58	1.50 ± 0.57	0.837
Self-worth	2.36 ± 0.49	2.36 ± 0.61	2.36 ± 0.54	0.997

The sample statistics presented in this table were mean ± standard deviation (SD) for continuous variables and frequency (percentage, %) for categorical variables. The listed *p* values of statistical tests were calculated using the Wilcoxon rank-sum test for continuous variables and the Fisher's exact test for categorical variables.

^∗^ *p* < 0.05, ^∗∗^*p* < 0.01, and ^∗∗∗^*p* < 0.001.

The article "Higher Rumination Tendency Is Associated with Reduced Positive Effects of Daily Activity Participation in People with Depressive Disorder" was published in 2022. Journal: Occup Ther Int.

**Table 3:** The differences in the profiles of participation restriction between participants with higher vs. lower rumination tendency.

Variable	Higher rumination	Lower rumination	Total	*p*
Types of participating restriction				0.445
Cultural activity	19 (22.35%)	11 (25.00%)	30 (23.26%)	0.827
Social activity	15 (17.65%)	11 (25.00%)	26 (20.16%)	0.359
Hobby activity	2 (2.35%)	1 (2.27%)	3 (2.33%)	1.000
Physical activity	5 (5.88%)	5 (11.36%)	10 (7.75%)	0.308
Health maintenance	6 (7.06%)	3 (6.82%)	9 (6.98%)	0.734
Home activity	15 (17.65%)	8 (18.18%)	23 (17.83%)	1.000
Vocational activity	23 (27.06%)	5 (11.36%)	28 (21.71%)	0.045^∗^
Missing	3	11	14	
Perceived reasons of restriction				0.009^∗∗^
Afraid of lonely/lack friends	2 (2.44%)	3 (6.98%)	5 (4.00%)	0.338
Poor ability	15 (18.29%)	3 (6.98%)	18 (14.40%)	0.111
Without family's support	29 (35.37%)	7 (16.28%)	36 (28.80%)	0.037^∗^
Poor economic resources	16 (19.51%)	10 (23.26%)	26 (20.80%)	0.648
Afraid of others' peculiar look	4 (4.88%)	2 (4.65%)	6 (4.80%)	1.000
Without enough time	6 (7.32%)	2 (4.65%)	8 (6.40%)	0.714
Poor health status	10 (12.20%)	14 (32.56%)	24 (19.20%)	0.009^∗∗^
Others	0 (0.00%)	2 (4.65%)	2 (1.60%)	0.113
Missing	6	12	18	
Expected involvement	2.57 ± 0.43	2.49 ± 0.55	2.55 ± 0.48	0.368
Negative affects due to restriction	2.06 ± 0.47	1.95 ± 0.59	2.02 ± 0.51	0.223

The sample statistics presented in this table were mean ± standard deviation (SD) for continuous variables and frequency (percentage, %) for categorical variables. The listed *p* values of statistical tests were calculated using the Wilcoxon rank-sum test for continuous variables and the Fisher's exact test for categorical variables.

^∗^ *p* < 0.05, ^∗∗^*p* < 0.01, and ^∗∗∗^*p* < 0.001.

## Data Availability

All required evidence that supports the results of this study has been reported. The other raw data could not be revealed or shared due to ethical concerns and the protection of participants' privacy.

## References

[1] World Health Organization Depression. http://www.who.int/mediacentre/factsheets/fs369/en/.

[2] American Psychiatric Association (2000). *Diagnostic and statistical manual of mental disorders*.

[3] Law M. (2002). Participation in the occupations of everyday life. *American Journal of Occupational Therapy*.

The article "Higher Rumination Tendency Is Associated with Reduced Positive Effects of Daily Activity Participation in People with Depressive Disorder" was published in 2022. Journal: Occup Ther Int.

[4] Wells K. B., Stewart A., Hays R. D. (1989). The functioning and well-being of depressed patients: results from the medical outcomes study. *JAMA*.

[5] Aneshensel D. S. (1985). The natural history of depressive symptoms: implications for psychiatric epidemiology. *Research in Community and Mental Health*.

[6] Keller M. B., Shapiro R. W., Lavori P. W., Wolfe N. (1982). Recovery in major depressive disorder: analysis with the life table and regression models. *Archives of General Psychiatry*.

[7] Nolen-Hoeksema S. (1991). Responses to depression and their effects on the duration of depressive episodes. *Journal of Abnormal Psychology*.

[8] Lyubomirsky S., Tkach C., Papageorgiou C., Wells A. (2004). The consequences of dysphoric rumination. *Depressive rumination: Nature, theory and treatment*.

[9] Donaldson C., Lam D. (2004). Rumination, mood and social problem-solving in major depression. *Psychological Medicine*.

[10] Lam D., Schuck N., Smith S., Farmer A., Checkley S. (2003). Response style, interpersonal difficulties and social functioning in major depressive disorder. *Journal of Affective Disorders*.

[11] Lyubomirsky S., Kasri F., Zehm K. (2003). Dysphoric rumination impairs concentration on academic tasks. *Cognitive Therapy and Research*.

[12] Nolen-Hoeksema S., Morrow J. (1991). A prospective study of depression and posttraumatic stress symptoms after a natural disaster: the 1989 Loma Prieta earthquake. *Journal of Personality and Social Psychology*.

[13] Huang L.-J., Wu C., Wu C.-H. (2015). Validation of the ruminative response scale-Chinese version (RRS-C) for persons with depression in Taiwan. *Taiwanese Journal of Psychiatry (Taipei)*.

[14] Lam D., Smith N., Checkley S., Rijsdijk F., Sham P. (2003). Effect of neuroticism, response style and information processing on depression severity in a clinically depressed sample. *Psychological Medicine*.

[15] Roberts J. E., Gilboa E., Gotlib I. H. (1998). Ruminative response style and vulnerability to episodes of dysphoria: gender, neuroticism, and episode duration. *Cognitive Therapy and Research*.

[16] Conway M., Csank P. A., Holm S. L., Blake C. K. (2000). On assessing individual differences in rumination on sadness. *Journal of Personality Assessment*.

[17] Segerstrom S. C., Tsao J. C., Alden L. E., Craske M. G. (2000). Worry and rumination: repetitive thought as a concomitant and predictor of negative mood. *Cognitive Therapy and Research*.

[18] Treynor W., Gonzalez R., Nolen-Hoeksema S. (2003). Rumination reconsidered: a psychometric analysis. *Cognitive Therapy and Research*.

[19] World Health Organization (2001). *International classification of functioning, disability and health*.

The article "Higher Rumination Tendency Is Associated with Reduced Positive Effects of Daily Activity Participation in People with Depressive Disorder" was published in 2022. Journal: Occup Ther Int.

[20] Huang L.-J., Wu C., Yeh H.-H., Huang P.-S., Yang Y.-H., Fang Y.-C. (2016). Mediation effects of daily activity participation between rumination and subjective quality of life in persons with depression. *Taiwanese Journal of Psychiatry (Taipei)*.

[21] Lepore S. J. (1997). Expressive writing moderates the relation between intrusive thoughts and depressive symptoms. *Journal of Personality and Social Psychology*.

[22] Morrow J., Nolen-Hoeksema S. (1990). Effects of responses to depression on the remediation of depressive affect. *Journal of Personality and Social Psychology*.

[23] Nolen-Hoeksema S., Wisco B. E., Lyubomirsky S. (2008). Rethinking rumination. *Perspectives on Psychological Science*.

[24] Beck A. T., Steer R. A., Brown G. K. (2000). *Manual for the Beck depression inventory-II*.

[25] American Psychiatric Association (1994). *Diagnostic and Statistical Manual of Mental Health Disorders*.

[26] Beck A. T., Steer R. A., Ball R., Ranieri W. F. (1996). Comparison of Beck depression inventories-IA and-II in psychiatric outpatients. *Journal of Personality Assessment*.

[27] Lu M.-L., Che H.-H., Chang S.-W., Shen W.-W. (2002). Reliability and validity of the Chinese version of the Beck depression inventory-II. *Taiwanese Journal of Psychiatry (Taipei)*.

[28] Wu C. Activity participation of people with schizophrenia: scale development and survey in Taiwan.

[29] Wu C.-H., Lee T.-H., Wu C. Measurement of activity participation among persons with schizophrenia living in the community.

[30] Linden M., Gehrke G., Geiselmann B. (2009). Profiles of recreational activities of daily living (RADL) in patients with mental disorders. *Psychiatria Danubina*.

[31] Nolen-Hoeksema S., Jackson B. (2001). Mediators of the gender difference in rumination. *Psychology of Women Quarterly*.

[32] Nolen-Hoeksema S., Aldao A. (2011). Gender and age differences in emotion regulation strategies and their relationship to depressive symptoms. *Personality and Individual Differences*.

[33] Kim S., Yu B. H., Lee D. S., Kim J. H. (2012). Ruminative response in clinical patients with major depressive disorder, bipolar disorder, and anxiety disorders. *Journal of Affective Disorders*.

[34] Chung M. S. (2014). Pathways between attachment and marital satisfaction: the mediating roles of rumination, empathy, and forgiveness. *Personality and Individual Differences*.

[35] James A., Wells A. (2003). Religion and mental health: towards a cognitive-behavioural framework. *British Journal of Health Psychology*.

[36] Flynn M., Kecmanovic J., Alloy L. B. (2010). An examination of integrated cognitive-interpersonal vulnerability to depression: the role of rumination, perceived social support, and interpersonal stress generation. *Cognitive Therapy and Research*.

The article "Higher Rumination Tendency Is Associated with Reduced Positive Effects of Daily Activity Participation in People with Depressive Disorder" was published in 2022. Journal: Occup Ther Int.

[37] Puterman E., DeLongis A., Pomaki G. (2010). Protecting us from ourselves: social support as a buffer of trait and state rumination. *Journal of Social and Clinical Psychology*.

[38] Christiansen C. H., Baum C. M., Christiansen C. H., Baum C. M. (1997). Understanding occupation: definitions and concepts. *Occupational Therapy: Enabling function and well-being*.

[39] Christiansen C. H. (1999). Defining lives: occupation as identity: an essay on competence, coherence, and the creation of meaning. *American Journal of Occupational Therapy*.

[40] Law M., Steinwender S., Leclair L. (1998). Occupation, health and well-being. *Canadian Journal of Occupational Therapy*.

[41] Magnus E. (2001). Everyday occupations and the process of redefinition: a study of how meaning in occupation influences redefinition of identity in women with a disability. *Scandinavian Journal of Occupational Therapy*.

[42] McIntosh W. D., Harlow T. F., Martin L. L. (1995). Linkers and nonlinkers: goal beliefs as a moderator of the effects of everyday hassles on rumination, depression, and physical Complaints1. *Journal of Applied Social Psychology*.

[43] Abramson L. Y., Metalsky G. I., Alloy L. B. (1989). Hopelessness depression: a theory-based subtype of depression. *Psychological Review*.

[44] Moberly N. J., Watkins E. R. (2010). Negative affect and ruminative self-focus during everyday goal pursuit. *Cognition and Emotion*.

[45] Gortner E. M., Rude S. S., Pennebaker J. W. (2006). Benefits of expressive writing in lowering rumination and depressive symptoms. *Behavior Therapy*.

[46] Sloan D. M., Marx B. P., Epstein E. M., Dobbs J. L. (2008). Expressive writing buffers against maladaptive rumination. *Emotion*.

[47] Gross J. J. (1999). Emotion regulation: past, present, future. *Cognition and Emotion*.

[48] Aldao A., Nolen-Hoeksema S., Schweizer S. (2010). Emotion-regulation strategies across psychopathology: a meta-analytic review. *Clinical Psychology Review*.

